The article "Assessment of Acupoint Therapy of Traditional Chinese Medicine on Cough Variant Asthma: A Meta-analysis" was retracted in 2024. Reasons: suspected computer-generated content; unreliable results or conclusions; concerns about the data; concerns about the results or conclusions.

# Assessment of Acupoint Therapy of Traditional Chinese Medicine on Cough Variant Asthma: A Meta-analysis

**DOI:** 10.1155/2022/4168308

**Published:** 2022-07-30

**Authors:** Hengjia Tu, Qingling Zhang

**Affiliations:** ^1^Nanshan School, Guangzhou Medical University, Guangzhou, 510000 Guangdong, China; ^2^State Key Laboratory of Respiratory Disease, National Clinical Research Center for Respiratory Disease, Guangzhou Institute of Respiratory Health, The First Affiliated Hospital of Guangzhou Medical University, Guangzhou, 510000 Guangdong, China

## Abstract

Acupoint application has been used in China to treat various illnesses for ages. In cough variant asthma (CVA), the main clinical sign is episodic night cough. Acupoint application therapy of traditional Chinese medicine is an effective procedure to treat cough variant asthma. The current study is designed to systematically assess the effectiveness of acupoint application therapy in traditional medicine for patients with cough variant asthma. The comprehensive computer retrieval related to comparison between acupoint application and nonacupoint application therapy for cough variant asthma was carried out in various databases (*n* = 8) from database establishment until July 4, 2021. Both English and Chinese articles about original investigations in humans were searched. Two independent authors extracted the data, and disagreements were resolved by discussion. ReviewManager 5.3 software provided by Cochrane did a meta-analysis of selected randomized controlled trials (RCTs). Quality of experimentation and risk bias were analyzed by the Cochrane Handbook tool. A total of thirteen randomized controlled clinical articles along with 1237 patients were included in the study. Findings of meta-analysis showed that compared with nonacupoint application treatment, the total effective rate of acupoint application treatment is more effective (RD = 0.13, 95% CI (0.09, 0.17), *Z* = 6.70, *P* < 0.00001). Besides, acupoint application can improve patients' lung function, the lung function index FVC (mean difference = 0.55, 95% confidence interval (0.42, 0.68), *Z* = 8.40, *P* < 0.00001), FEV1 (MD = 0.35, 95% CI (0.23, 0.47), *Z* = 5.86, *P* < 0.00001), *FEV1/FVC (%)* (MD = 12.68, 95% CI (4.32, 21.03), *Z* = 2.97, *P* = 0.003), *FEV1 (%)* (MD = 8.63, 95% CI (8.01, 9.25), *Z* = 27.44, *P* < 0.00001), and *PEF (day)* (MD = 0.62, 95% CI (0.52, 0.71), *Z* = 12.40, *P* < 0.00001) of patients treated by acupoint application therapy were increased. Moreover, acupoint application might lower the level of immunoglobulin E (MD = −54.58, 95% CI (−63.54, −45.61), *Z* = 11.93, *P* < 0.00001) and EOS (MD = −0.21, 95% CI (−0.35, −0.06), *Z* = 2.77, *P* = 0.006). The LCQ (Leicester cough questionnaire) total score of CVA patients was also increased (MD = 2.30, 95% CI (1.55, 3.06), *Z* = 5.98, *P* < 0.00001). Acupoint application therapy is effective in controlling symptoms of CVA. It also has a positive effect in improving lung function and life quality of patients. It can reduce the eosinophil levels and peripheral blood IgE levels of patients as well.

## 1. Introduction

Cough variant asthma (CVA) is a particular form with typical common cold symptoms and dry, nonproductive cough. Other manifestations, like dyspnea or gasping, are not generally observed; however, there could be episodic night cough which can be alleviated by a bronchodilator [1]. The symptoms of chronic cough in CVA might result in physiological disorders, psychological nervousness, and disruption of the socialization process. Previous findings revealed that persistent cough is the main risk factor (32.6%) of CVA in five territories of the Chinese Republic [2].

In addition, the prevalence of cough variant asthma is still prominent due to air pollution [3], smoking, allergens, and other reasons.

Current treatments for CVA are generally the same as ordinary respiratory illness, along with bronchodilators, glucocorticoid drugs, antihistamines, and leukotriene receptor antagonists [4]. Although these medications effectively control CVA symptoms and regulate inflammatory responses, the course of treatment is often long, and the patient's long-term compliance with medication is unwarranted. At the same time, some drugs will also cause osteoporosis [5], induce tissue degeneration, and other adverse reactions.

Acupoint application (AP) is a traditional Chinese medicine (TCM) method with a long history. The main steps of this treatment are grinding the herbs into powder and turning them into herbal patches, directly sticking to acupoints or affected areas to treat chronic cough. Studies have shown that acupoint application can affect the level of immunoglobulin and eosinophils in patients with CVA, regulate the proportion of lymphocytes, and influence the proportion of some cytokines, such as TGF, TNF, and IF, to control the symptoms of CVA and achieve long-term relief [6–8].

Recently, there have been many studies demonstrating AP's positive results for curing CVA [9]. However, those studies are limited to a few parameters and have a small sample size. Similarly, few researchers have conducted a systematic literature review of acupoint application in children [10]. Still, those studies have limited findings and mainly focus on only children. We, therefore, systemically searched and analyzed the consequences of stimulating acupoints for the cure of cough variant asthma through the available literature from several databases. Randomized controlled trials have been conducted comparing AP-based treatment with non-AP-based treatments. Results have been assessed based on quality and probability of biasness after consulting the Cochrane Handbook [11].

## 2. Methodology

### 2.1. Search Strategy

We systematically searched the literature for the formation of every database to July 4, 2021. Databases include PubMed (https://pubmed.ncbi.nlm.nih.gov/), EMBASE (https://www.embase.com/landing?status=grey), Web of Science (https://mjl.clarivate.com/search-results), the Cochrane Library (https://www.cochranelibrary.com/), Chinese Journal Full-Text Database (CNKI) (http://kns55.en.eastview.com/kns55/brief/result.aspx?dbPrefix=CJFD), Database of Chinese Sci-Tech Periodicals (VIP) (http://www.nlc.cn/newen/periodicals/), “Wanfang” Database (http://www.wanfangdata.com/), and China Biology Medicine Disc (CBM)(http://allie.dbcls.jp/pair/CBM;Chinese+BioMedical+Disc.html). The following keywords were used: “stimulating acupoints,” “acupoint sticking,” “traditional Chinese medicine,” “TCM,” “acupoint,” “CVA,” “cough variant asthma,” “cough type asthma,” “cough-variant asthma,” “randomized controlled trial,” “random,” “control and trial,” and “RCT.”

The search methodology for PubMed is mentioned below:

The following terms were applied: Medicine, Chinese Traditional [MeSH Terms]) OR Traditional Chinese Medicine[MeSH Terms]) OR Chinese Traditional Medicine[MeSH Terms]) OR acupuncture[Abstract]) OR moxibustion[Abstract]) OR “auricular points plaster therapy”[Abstract]) OR “acupoint sticking”[Abstract])) AND “Cough Type Asthma”[Abstract]) OR “Cough variant asthma”[Abstract]) OR “Cough-Type Asthma”[Abstract]) OR “Cough-variant asthma”[Abstract]).

#1 “auricular points plaster therapy”[Abstract/Title].

#2 “acupoint sticking”[Abstract/Title]).

#3 Traditional Chinese Medicine[MeSH Terms].

#4 “ #1 OR #2 OR #3 ”.

#5 “Cough Type Asthma”[Abstract/Title].

#6 “Cough variant asthma”[Abstract/Title].

#7 “Cough-variant asthma”[Abstract/Title].

#8 “CVA” [Abstract/Title].

#9 “ #5 OR #6 OR #7 OR #8”.

#10 “Randomized controlled trial”[Abstract/Title].

#11 “Random”[Abstract/Title].

#12 “Control”[Abstract/Title].

#13 “Trial”[Abstract/Title].

#14 “ #10 OR #11 OR #12 OR #13”.

#15 “ #4 AND #9 AND 14”.

Moreover, to include all the possible information, incomplete and finished experiments on the Chinese Scientific Experiments Register (update to July 2021) and World Health Organization ICTRP (http://www.who.int/ictrp/en/) were also explored.

### 2.2. Study Selection

#### 2.2.1. Inclusion Standard for Literature

1. Randomized controlled trials on acupoint application on ACV were applied
2. Languages were only Chinese and English
3. By using the proper standard of diagnosis, individuals were evaluated as patients with CVA
4. From the already published information, the interference criteria for the test sample was acupoint application/acupoint application with a combination of other treatment methods. However, in the control group, no acupoint application treatment was included; e.g., data from Western medicine or traditional Chinese medicine were included in the control group
5. In similar research, when the test set was an acupoint application connected with different treatment strategies, with inference criteria utilized by the control set, it is necessary that only AP interference is similar to the experimental dataset

#### 2.2.2. Literature Exclusion Standard

1. Items considered for exclusion were meeting recordings, theoretical research, case studies, and brief information experience of experts. These were not included
2. Repeatedly published information was excluded from this study
3. Articles not using the proper standard of diagnosis of CVA were also not included
4. Data about the trials on animals
5. Trials that were not properly controlled without clinical manifestation were not taken for this study
6. Incomplete literature data
7. Obvious errors such as self-contradiction and fabricating data were also excluded

### 2.3. Data Extraction and Management

From published articles, the study plan section was screened in the following manner: time of research, methodology, and blinding (including allocation concealment, blinding of research volunteers, health professionals, and assessment of results). These parameters were studied and included in the analysis.

From the studied sections, participants of those studied articles were also screened. The following features of the study participants, age limit, gender, disease identification, other signs, and treatment count, as well as control samples, key features of treatment and control groups, and total completed experiments as well as incomplete or withdrawn, were taken for further analysis.

In interventions, site for acupoint application, time of interference, and noninterference were focused.

From the results section of the literature, total effective rate, forced expiratory volume (FVC), forced expiratory volume in one second, FEV1/FVC (%), FEV1/predication (FEV1/pre), peak expiratory flow (PEF), EOS count per milliliter in peripheral blood, IgE level per milliliter in the peripheral blood, and LCQ total score were taken for further study and analysis.

### 2.4. Quality Assessment

Evaluation of standard of research was done by ReviewManager 5.3 software risk bias assessment tool equipped from Cochrane Collaboration: (a) to generate the randomized data, (b) concealing the allocation, (c) blinding of research individuals, (d) blinding of the evaluation of results, (e) no proper information retrieved, (f) prediction of specific results, and (g) different partialities. Each group was regarded as “high risk of bias” and “low risk of bias”/“unclear risk of bias.”

### 2.5. Statistical Analysis

We used the Cochrane ReviewManager 5.3 software for meta-analysis and assessment of reviewed data. Dichotomous data were displayed as odds ratio/risk ratio having 95% confidence intervals that predict the chance of risk or relative risk. Continuous variable dataset assessment was done by MD odds ratio and 95% confidence intervals (CIs). Key point of evaluation is the research volunteers.

Assessment of the experiments was done for clinical heterogeneity (demographic features, features of ailments, and therapies), diversity in methodology (planning, execution, and risk of bias), and statistical diversity. The chi-square test was applied with a *P* value: if *P* value was less than 0.10, this showed statistically significant results. *I*^2^ statistic was applied as guided by the Cochrane Handbook for Systematic Reviews of Interventions. If*I*-square (*I*^2^) was used as a statistical method to assess data heterogeneity, the value of *I*^2^ < 40% was indicative of less heterogeneity, whereas more than 75% indicated significant heterogeneity in experimentation. The funnel plot visually analyzed the “risk of reporting” bias.

Sensitivity analysis was done as described below: assessment of outcomes of two statistical models, i.e., random-effect model (REM) and fixed model, were applied and compared. If *I*^2^ > 50%, the random-effect model (REM) was applied for assessment.

## 3. Results

### 3.1. Literature Survey

A total of 534 records were analyzed after excluding the duplicated data. This data was further meta-analyzed, and all the information related to the search for knowledge and protocol selection for research is presented in Figure 1.

### 3.2. Key Features of the Research

Out of the screened articles, thirteen articles were disclosed in 2014-2020 from nine provinces in China about AP in CVA. A total of 1237 volunteers participated in these researches, aged of 4-65 years. In previously published articles, the test groups consisted of patients who had undergone AP along with different treatments. In the control group, no AP was applied, and only Western or traditional Chinese medicines were used for the treatment of CVA.

The acupoint application test and control samples had 621 and 616 cases, respectively. Key features of all elected research are mentioned in Table 1.

### 3.3. Risk of Bias

Assessment of “risk of bias” is presented in Figure 2. Seven types of research were examined with minimum risk of bias in the assembly of randomly generated sequences, and other studies showed no precise results. Out of screened articles, six were found to carry a low risk of bias in allocation concealment, and others had an uncertain risk of bias in it. All other findings of articles were categorized based on higher risk. The selected researches showed a low risk of bias related to the incomplete dataset, SOR, and other biases.

### 3.4. Analysis of Total Effective Rate of Acupoint Application Therapy for Cough Variant Asthma

The sum of eleven types of research [9, 12–21] included 1043 participants who described total effective rates (Table 2). Heterogeneity among datasets was chi^2^ = 11.37, *P* = 0.33, and *I*^2^ = 12%, and the fixed-effect model was applied for evaluation (Figure 3). Total effective rate of CVA treatment in the experimental group was more effective than that in the control group (RD = 0.13, 95% confidence interval (0.09, 0.17), *Z* = 6.70, *P* < 0.00001). The funnel plot revealed a uniform plot on both sides (left and right) and stacked on the upper side, showing a certain risk of bias, as shown in Figure 4.

### 3.5. Analysis of Lung Function Index in Acupoint Application Treatment of CVA

#### 3.5.1. Analysis of Lung Function Index FVC in Acupoint Application Therapy of Cough Variant Asthma

Three articles [14, 16, 18] reported lung function index FVC (Table 3). We used a randomized-effect analysis that analyzed the cumulative impact of the amount of research, indicating that acupoint application treatment was more effective to the experimental set to improve lung function index FVC (MD = 0.55, 95% CI (0.42, 0.68), *Z* = 8.40, *P* < 0.00001) (Figure 5)

#### 3.5.2. Assessment of Pulmonary Function Index FEV1 in Acupoint Application Therapy of Cough Variant Asthma

Five articles [12, 14, 16, 18, 22] described cough variant asthma pulmonary function measure FEV1 with acupoint application therapy (Table 4), in the case of 597 cases. The random-effect analysis model was applied for analysis (mean difference = 0.35, 95% confidence interval (0.23, 0.47), *Z* = 5.86, *P* < 0.00001). These findings suggested that AP has more ability to improve the pulmonary function index FEV1 compared to the control group (Figure 6). A test evaluated heterogeneity in research (*P* = 0.003, *I*^2^ = 76%), and a subgroup analysis was performed. In the subgroup of patients younger than 7, the subgroup evaluation of four researchers reported a statistically small difference (mean difference = 0.30, 95% confidence interval (0.22, 0.37), *Z* = 8.00, *P* < 0.00001). In the subgroup of patients older than 7, the subgroup analysis showed a statistically significant difference (MD = 0.57, 95% CI (0.41, 0.73), *Z* = 6.93, *P* < 0.00001).

#### 3.5.3. Assessment of Pulmonary Function Index FEV1/FVC (%) in Acupoint Application Therapy of Cough Variant Asthma

Three types of research [14, 16, 22] with 432 patients evaluated CVA pulmonary function indicator FEV1/FVC (%) of acupoint application therapy (Table 5). The random-effect analysis model was applied for analysis (MD = 12.68, 95% CI (4.32, 21.03), *Z* = 2.97, *P* = 0.003). This suggests that acupoint application improves pulmonary function index FEV1/FVC (%) better than the control group. Heterogeneity among researchers (*P* < 0.00001, *I*^2^ = 98%) and subgroup analysis were performed. For the subgroup of patients whose intervention period is less than 30 days, subgroup evaluation in the 180 patients resulted in a statistically significant difference (MD = 5.05, 95% CI (3.30, 6.80), *Z* = 5.65, *P* < 0.00001). Statistically significant results were found in those patients (*n* = 120) whose intervention period was more than 30 days and less than 6 months (MD = 14.66, 95% CI (12.27, 17.05), *Z* = 12.00, *P* < 0.00001), whereas 120 patients were found with statistically significant results whose intervention period was more than 6 months (MD = 18.45, 95% CI (15.81, 21.09), *Z* = 13.72, *P* < 0.00001) (Figure 7).

#### 3.5.4. Analysis of the Pulmonary Function Index FEV1 (%) in Acupoint Application Therapy of Cough Variant Asthma

The fixed-effect model showed that AP treatment was more effective for the experimental group for improving lung function index FEV1 (%) (MD = 8.63, 95% CI (8.01, 9.25), *Z* = 27.44, *P* < 0.00001). The difference between the three subgroups was significantly small (*I*^2^ = 0%) (Table 6, Figure 8).

#### 3.5.5. Analysis of the Pulmonary Function Index PEF (day) for Acupoint Application Therapy of Cough Variant Asthma

Three screened reports [16, 18, 22] reported lung function index PEF (day) (Table 7) of 336 patients. A fixed-effect model was applied for analysis of the cumulative impact of the amount of experiment (mean difference = 0.62, 95% analysis of confidence interval (0.52, 0.71), *Z* = 12.40, *P* < 0.00001) which demonstrated that AP treatment is more effective in improving the pulmonary function index PEF compared to the control group (Figure 9).

### 3.6. Analysis of the Laboratory Indices in Acupoint Application Treatment of CVA

#### 3.6.1. Analysis of the Peripheral Blood IgE Level in Acupoint Application Treatment of CVA

Few studies [13, 16, 18, 19, 22] reported the peripheral blood IgE level as a measure of cough variant asthma for the acupoint application therapy (Table 8). This was observed in almost 522 cases. The fixed-effect analysis model was applied to analyze two groups of samples (MD = −54.58, 95% CI (−63.54, −45.61), *Z* = 11.93, *P* < 0.00001), which reported that acupoint application treatment could better decrease the peripheral blood IgE level of CVA patients as compared to control samples (Figure 10).

#### 3.6.2. Analysis of the Peripheral Blood Eosinophilic Granulocyte (EOS) Count in Acupoint Application Treatment of CVA

Two studies [16, 18] reported peripheral blood EOS count (∗10^9^/L), the cough variant asthma measure for acupoint application therapy (Table 9), with the sum of 204 cases. Heterogeneity analysis evaluated significant homogeneity in research (*I*^2^ = 66%). The random-effect analysis algorithm was applied to analyze two groups of samples (MD = −0.21, 95% CI (−0.35, −0.06), *Z* = 2.77, *P* = 0.006), indicating that acupoint application treatment could better decrease the peripheral blood EOS count of CVA patients as compared to control samples (Figure 11).

### 3.7. Analysis of the LCQ Score in Acupoint Application Treatment of CVA

Two studies [20, 23] reported LCQ scores, having a total of 152 cases. Heterogeneity analysis reported a small homogeneity in the research (*I*^2^ = 0%) (Table 10). The fixed-effect analysis model was applied to analyze the 2 groups of samples (MD = 2.30, 95% CI (1.55, 3.06), *Z* = 5.98, *P* < 0.00001), evaluating acupoint application treatment which might lead to better increase of the LCQ score of CVA patients compared with the control group (Figure 12).

## 4. Discussion

It is widely believed that CVA is regarded as a particular form of respiratory illness with a histopathological process, just like common asthma. These include hyperresponsiveness (BHR), eosinophilic airway inflammation, and airway remodeling [24]. Various inflammatory cells, including eosinophils, neutrophils, and mastocytes, interact with cytokines and inflammatory mediators to form a complex immune network and form chronic nonspecific inflammation in this disorder, indirectly showing characteristic BHR, cough receptor hypersensitivity, inflammatory cell infiltration, and cells having genes expressed for inflammation [25]. This histopathological process leads to chronic cough, which is common in clinical practice. CVA may also be transformed into typical asthma.

Asthma can be treated by inhaled glucocorticoids and leukotriene modulator drugs, etc. These drugs are categorized into a control group and need to be taken for a long period for the therapy to be effective, whereas other drugs include palliative drugs which include short-acting 13*β*_2_ receptor agonists, inhaled anticholinergic drugs, and short-acting theophylline. These drugs are very effective in alleviating symptoms, reducing airway inflammation, and improving quality of life. However, adverse reactions of these drugs have also been observed. Glucocorticoids may cause hoarseness of voice and oral candida infection. The use of *β* receptor agonists may lead to sympathetic nerve excitation and accelerated heart rate, resulting in palpitations, chest pain, and other symptoms. So, it is advised to use these drugs only in emergencies and for the shorter period of time. Acupoint application is a nice alternative to these drugs [26].

Acupoint sticking therapy has a long history in traditional Chinese medicine. The main steps of this treatment are as follows. First, a variety of herbs were ground into a powder. Second, adhesive materials such as ginger water were prepared. Next, mix the powder with the adhesive to make a pulp salve that may look like “caking agent” and put it on certain acupuncture points of the body. For treating cough variant asthma, we often choose the “TianTu” (RN22), “DaZhui”(DU14), “FeiShu”(BL13), and “ShanZhong” (RN17) acupoints. Acupoint application allows drugs to be absorbed directly through the skin into capillaries without the need for liver metabolism, which preserves the biological activity of some drugs [7, 8].

Acupoint application has an advantage over other treatment therapies in treating asthma as acupoint stimulation promotes flow of blood to dispel pathogenic factors. This can stimulate the body's immunity and reduce allergic states [27]. But still, no fully revealed mechanism of acupoint application has been observed in the treatment of cough variant asthma. IgE forms a complex immune interaction with various inflammatory factors like IL-4, IgA, IgE, and IgG to alleviate the symptoms of cough variant asthma [28]. So, it is suggested that the acupoint procedure can treat the CVA via regulating the inflammatory mediators [29].

Findings of this meta-analysis revealed that the rate of effectiveness, lung function index (FVC, FEV1, FEV1/FVC (%), FEV1 (%), PEF (day)) of the CVA sample showed more significant values as compared to the control group, whereas IgE and peripheral blood EOS count showed lower values when compared with control samples. This suggested that AP for cure of CVA has better efficacy than the other drug treatments.

The main advantage of this study is that we conducted a meta-analysis of 13 RCTs involving 1237 participants. Compared to previous systematic reviews of acupoint application for CVA [30], this study included a larger sample size and included age groups including infants, children, and the elderly. In addition, differences in clinical response rate, lung function, LCQ scores, and some biochemical blood indicators were investigated.

However, this study still has some limitations. The foremost limitation is that, although the treatment of CVA by acupoint application is frequently used, random clinical controlled studies are usually single-center studies with a small sample size. There are problems such as having no recognized standard for efficacy evaluation and clinical heterogeneity. These problems suggest the need for high-quality clinical research methods in treating CVA by acupoint application, including correct randomization, double-blind, and allocation concealment methods, as well as large-scale multicenter studies. Second, since the acupoint application requires the application operating on the patient, and the herbs have a special smell, it is impossible to blind the patients during the operation in all employed research. Therefore, based on risk-of-bias assessment software provided by the Cochrane Organization, the “blinding of participants and personnel” in whole reports was evaluated as “high risk.” Third, the language of retrieval in the present research was in Chinese and English, and the literature was only from 8 databases. Besides, all the reports used in the meta-analysis were in Chinese, and all the experiments were conducted in China, limiting the present results' specifications because of sample features. Fourth, due to the complexity of acupoint application, this study mainly focused on the treating method of acupoint application but did not explore the influence of different acupoint selections and the type of herbal medicine on treating effectiveness.

## 5. Conclusion

The current study concluded that acupoint application is better for the CVA treatment than the control group, which was treated with other traditional medicines. Moreover, it was observed that AP improved respiration and chronic airway inflammation by reducing eosinophil levels and peripheral blood IgE levels.

## Figures and Tables

**Figure 1:** The process of literature search and study selection for the research.

**Figure 2:** Assessment of the risk of bias of different research articles.

**Figure 3:** Analysis of the total effective rate for acupoint application therapy for CVA.

**Figure 4:** The funnel plot of the analysis of the total effective rate to show the risk of bias.

**Figure 5:** Analysis of lung function index FVC, which shows the effectiveness of acupoint application treatment in the experimental group.

**Figure 6:** Analysis of the lung function index FEV1 through random-effect analysis model.

**Figure 7:** Analysis of the lung function index FEV1_FVC (%), which shows the improvement in lung function due to AP.

**Figure 8:** Analysis of the lung function index FEV1 (%) by fixed-effect model.

**Figure 9:** Analysis of the lung function index PEF to evaluate the cumulative effect of the AP treatment.

**Figure 10:** Analysis of the peripheral blood IgE level in patients suffering from CVA treated with acupoint application therapy.

**Figure 11:** Heterogeneity analysis of the EOS count to evaluate the homogeneity of research.

**Figure 12:** Heterogeneity analysis of the LCQ score of acupoint application.

**Table 1:** Characteristics of studies.

Study	Number of patients		Age	Gender (male/female)	Interventions	Control group	Intervention duration (day)	Outcome assessment	Length of follow-up	Region
	Intervention group	Control group								
Yu Tong 2017	41	40	5.94 ± 1.28	45/36	Acupoint application+normal treatment	(1)	30	1, 2	6 months	Zhejiang, China
Xue Ming 2018	45	45	6.54 ± 2.1	46/44	Acupoint application+normal treatment	(2)	30	1, 5	Not mentioned	Shanxi, China
Ma Ying 2018	66	66	4.77 ± 1.31	65/67	Acupoint application+normal treatment	(1)	365	2, 4	1 year	Henan, China
Wang Long 2017	25	25	40.41 ± 6.39	20/30	Acupoint application+normal treatment	(2)	28	1	Not mentioned	Liaoning, China
Gao Xiyue 2017	31	31	8.95 ± 2.13	34/28	Acupoint application+normal treatment	(1)	30	6	3 months	Sichuan, Chian
Ye Jianlin 2017	90	90	6.35 ± 2.27	96/84	Acupoint application+normal treatment	(2)	28	1, 2	Not mentioned	Guangdong, China
Li Limei 2019	30	30	5.62 ± 1.33	33/27	Acupoint application+normal treatment	(1)	90	1	Not mentioned	Guangdong, China
Li Qiaoxiang 2017	60	60	7.28 ± 4.75	58/62	Acupoint application+normal treatment	(1)	45	1, 2, 3, 4	Not mentioned	Hunan, China
Tang Jianwen 2015	48	48	64.05 ± 8.70	54/42	Acupoint application+normal treatment	(3), (4)	30	1, 2	Not mentioned	Jiangsu, China
Zhao Qi 2018	42	42	6.13 ± 2.09	52/32	Acupoint application+normal treatment	(8)	28	1, 2, 3, 4	Not mentioned	Sichuan, Chian
Zhang Xiaoyan 2014	50	46	4.65 ± 1.60	55/41	Acupoint application+normal treatment	(5), (6)	30	1 + 4	Not mentioned	Hebei, China
Gou Li 2020	45	45	8.80 ± 0.80	44/46	Acupoint application+normal treatment	(1), (7)	28	1, 6	Not mentioned	Henan, China
Sui Aifeng 2015	48	48	65.31 ± 10.49	47/49	Acupoint application+normal treatment	(3), (4)	1095	1, 2	Not mentioned	Liaoning, China

Notes: (1) montelukast, (2) aminophylline, (3) salmeterol, (4) fluticasone propionate, (5) ketotifen, (6) procaterol, (7) budesonide, (8) salbutamol. 1: total effective rate; 2: lung functions (FVC, FEV1,FEV1/FVC, FEF, and PEF); 3: the peripheral blood eosinophil (EOS) count; 4: peripheral blood IgE content; 5: asthma control test(ACT) score; 6: Leicester cough questionnaire (LCQ).

**Table 2:** Evaluation of total effective rate by chi-square and fixed effect model.

Study or subgroup	Experimental		Control		Weight	Risk Difference
	Events	Total	Events	Total		M-H, fixed, 95% CI
Gou Li 2020	45	45	43	45	8.6%	0.04 [-0.03, 0.12]
Li Limei 2019	29	30	21	30	5.8%	0.27 [0.09, 0.44]
Li Qiaoxiang 2017	58	60	52	60	11.5%	0.10 [0.00, 0.20]
Sui Aifeng 2015	45	48	37	48	9.2%	0.17 [0.03, 0.30]
Tang Jianwen 2015	45	48	37	48	9.2%	0.17 [0.03, 0.30]
Wang Long 2017	22	25	18	25	4.8%	0.16 [-0.06, 0.38]
Xue Ming 2018	41	45	39	45	8.6%	0.04 [-0.09, 0.17]
Ye Jianlin 2017	85	90	75	90	17.3%	0.11 [0.02, 0.20]
Yu Tong 2017	38	41	30	40	7.8%	0.18 [0.02, 0.33]
Zhang Xiaoyan 2014	47	50	37	46	9.2%	0.14 [0.00, 0.27]
Zhao Qi 2018	40	42	33	42	8.1%	0.17 [0.03, 0.31]
Total (95% CI)		524		519	100%	0.13 [0.09, 0.17]
Total events	495		422			

Heterogeneity: chi^2^ = 11.37; df = 10 (*P* = 0.33); *I*^2^ = 12%. Test for overall effect: *Z* = 6.70 (*P* < 0.00001).

**Table 3:** FVC index of control and experimental groups to analyze the cumulative effect of research.

Study or subgroup	Mean	Experimental		Mean	Control		Weight	Mean difference
		SD	Total		SD	Total		IV, random, 95% CI
Li Qiaoxiang 2017	4.04	0.49	60	3.45	0.57	60	27.0%	0.59 [0.40, 0.78]
Ye Jianlin 2017	3.83	0.54	90	3.4	0.47	90	35.3%	0.43 [0.28, 0.58]
Zhao Qi 2018	3.2	0.31	42	2.57	0.33	42	37.8%	0.63 [0.49, 0.77]
Total (95% CI)			192			192	100%	0.55 [0.42, 0.68]

Heterogeneity: tau^2^ = 0.01; chi^2^ = 4.01; df = 2 (*P* = 0.13); *I*^2^ = 50%. Test for overall effect: Z = 8.40 (*P* < 0.00001).

**Table 4:** Analysis of the lung function index FEV1 which shows statistically significant differences among subgroups.

Study or subgroup	Mean	Experimental		Mean	Control		Weight	Mean difference
		SD	Total		SD	Total		IV, random, 95% CI
1.3.1 age ≤ 7								
Ma Ying 2018	1.39	0.11	66	1.12	0.12	66	29.0%	0.27 [0.23, 0.31]
Ye Jianlin 2017	2.6	0.43	90	2.2	0.36	90	23.2%	0.40 [0.28, 0.52]
Yu Tong 2017	1.77	0.43	41	1.54	0.47	40	16.3%	0.23 [0.03, 0.43]
Zhao Qi 2018	3.32	0.62	42	3.05	0.58	42	12.3%	0.27 [0.01, 0.53]
Subtotal total (95% CI)			239			238	80.8%	0.30 [0.22, 0.37]
Heterogeneity: tau^2^ = 0.00; chi^2^ = 4.62; df = 3 (*P* = 0.20); *I*^2^ = 35% Test for overall effect: *Z* = 8.00 (*P* < 0.00001)								
1.3.2 age > 7								
Li Qiaoxiang 2017	3.22	0.43	60	2.65	0.47	60	19.2%	0.57 [0.41, 0.73]
Subtotal Total (95% CI)			60			60	19.2%	0.57 [0.41, 0.73]
Heterogeneity: not applicable Test for overall effect: *Z* = 6.93 (*P* < 0.00001)								
Total (95% CI)			299			298	100%	0.35 [0.23, 0.47]

Heterogeneity: tau^2^ = 0.01; chi^2^ = 16.35; df = 4 (*P* = 0.003); *I*^2^ = 76%. Test for overall effect: *Z* = 5.86 (*P* < 0.00001). Test for subgroup difference: chi^2^ = 9.09; df = 1 (*P* = 0.003); *I*^2^ = 89.0%.

**Table 5:** Evaluation of effectiveness of acupoint application treatment on lung function of various groups of the research participants.

Study or subgroup	Mean	Experimental		Mean	Control		Weight	Mean difference
		SD	Total		SD	Total		IV, random, 95% CI
1.4.1 intervention period≤30 days								
Ye Jianlin2017	62.76	6.41	90	57.71	5.54	90	33.7%	5.05 [3.30, 6.80]
Subtotal total (95% CI)			90			90	33.7%	5.05 [3.30, 6.80]
Heterogeneity: not applicable Test for overall effect: *Z* = 5.65 (*P* < 0.00001)								
1.4.2 intervention period > 30 days and intervention period ≤ 6 months								
Li Qiaoxiang 2017	76.99	7.24	60	62.33	6.09	60	33.3%	14.66 [12.27, 17.05]
Subtotal total (95% CI)			60			60	33.3%	14.66 [12.27, 17.05]
Heterogeneity: not applicable Test for overall effect: *Z* = 12.00 (*P* < 0.00001)								
1.4.3 intervention period > 6 months								
Ma Ying 2018	80.78	8.11	66	62.33	7.32	66	33.1%	18.45 [15.81, 21.09]
Subtotal total (95% CI)			66			66	33.1%	18.45 [15.81, 21.09]
Heterogeneity: not applicable Test for overall effect: *Z* = 13.72 (*P* < 0.00001)								
Total (95% CI)			216			216	100%	12.68 [4.32, 21.03]

Heterogeneity: tau^2^ = 53.16; chi^2^ = 83.74; df = 2 (*P* < 0.00001); *I*^2^ = 98%. Test for overall effect: *Z* = 2.97 (*P* = 0.003). Test for subgroup difference: chi^2^ = 83.74; df = 2 (*P* < 0.00001); *I*^2^ = 97.6%.

**Table 6:** Evaluation of effectiveness of AP therapy through pulmonary function index % through fixed-effect model.

Study or subgroup	Mean	Experimental		Mean	Control		Weight	Mean difference
		SD	Total		SD	Total		IV, fixed, 95% CI
Sui Aifeng 2015	79.28	2.1	48	70.65	2.25	48	50.1%	8.63 [7.76, 9.50]
Tang Jianwen 2015	79.29	2.1	48	70.66	2.26	48	49.9%	8.63 [7.76, 9.50]
Total (95% CI)			96			96	100%	8.63 [8.01, 9.25]

Heterogeneity: chi^2^ = 0.00; df = 1 (*P* = 1.00); *I*^2^ = 0%. Test for overall effect: *Z* = 27.44 (*P* < 0.00001).

**Table 7:** Analysis of pulmonary function index (day) of three screened reports through fixed-effect model.

Study or subgroup	Mean	Experimental		Mean	Control		Weight	Mean difference
		SD	Total		SD	Total		IV, fixed, 95% CI
Li Qiaoxiang 2017	3.42	0.87	60	2.91	0.44	60	15.6%	0.51 [0.26, 0.76]
Ma Ying 2018	3.32	0.31	66	2.67	0.33	66	79.6%	0.65 [0.54, 0.76]
Zhao Qi 2018	6.36	1.03	42	5.95	1.04	42	4.8%	0.41 [-0.03, 0.85]
Total (95% CI)			168			168	100%	0.62 [0.52, 0.71]

Heterogeneity: chi^2^ = 1.91; df = 2 (*P* = 0.38); *I*^2^ = 0%. Test for overall effect: *Z* = 12.40 (*P* < 0.00001).

**Table 8:** Level of IgE in peripheral blood as a measure of CVA.

Study or subgroup	Mean	Experimental		Mean	Control		Weight	Mean difference
		SD	Total		SD	Total		IV, fixed, 95% CI
Li Qiaoxiang 2017	119.33	79.63	60	167.94	89.23	60	8.8%	-48.61 [-78.87, -18.35]
Ma Ying 2018	131.2	26.4	66	189.3	31.7	66	81.2%	-58.10 [-68.05, -48.15]
Xue Ming 2018	124.24	112.45	45	171.58	112.99	45	3.7%	-47.34 [-93.92, -0.76]
Zhang Xiaoyan 2014	136.61	115.56	50	158.94	127.27	46	3.4%	-22.33 [-71.10, 26.44]
Zhao Qi 2018	134.61	117.61	42	156.49	124.88	42	3.0%	-21.88 [-73.76, 30.00]
Total (95% CI)			263			259	100%	-54.58 [-63.54, -45.61]

Heterogeneity: chi^2^ = 3.93; df = 4 (*P* = 0.42); *I*^2^ = 0%. Test for overall effect: *Z* = 11.93 (*P* < 0.00001).

**Table 9:** Decrease in peripheral blood EOS count of experimental samples as compared to control samples.

Study or subgroup	Mean	Experimental		Mean	Control		Weight	Mean difference
		SD	Total		SD	Total		IV, random, 95% CI
Li Qiaoxiang 2017	1.09	0.33	60	1.23	0.21	60	55.4%	-0.14 [-0.24, -0.04]
Zhao Qi 2018	0.64	0.24	42	0.93	0.39	42	44.6%	-0.29 [-0.43, -0.15]
Total (95% CI)			102			102	100%	-0.21 [-0.35, -0.06]

Heterogeneity: tau^2^ = 0.01; chi^2^ = 2.98; df = 1 (*P* = 0.08); *I*^2^ = 66%. Test for overall effect: *Z* = 2.77 (*P* = 0.006).

**Table 10:** Fixed-effect model analysis which shows increase in LCQ score.

Study or subgroup	Mean	Experimental		Mean	Control		Weight	Mean difference
		SD	Total		SD	Total		IV, fixed, 95% CI
Gao Xiyue 2017	15.7	2.18	30	13.25	2.83	32	36.3%	2.45 [1.20, 3.70]
Gou Li 2020	18.06	2.53	45	15.84	2.02	45	63.7%	2.22 [1.27, 3.17]
Total (95% CI)			75			77	100%	2.30 [1.55, 3.06]

Heterogeneity: chi^2^ = 0.08; df = 1 (*P* = 0.77); *I*^2^ = 0%. Test for overall effect: *Z* = 5.98 (*P* < 0.00001).

## Data Availability

The data are available from the corresponding author upon reasonable request.
